The article "Running Against the Wnt: How Wnt/β-Catenin Suppresses Adipogenesis" was published in 2021. Journal: Front Cell Dev Biol.

# Running Against the Wnt: How Wnt/β-Catenin Suppresses Adipogenesis

**DOI:** 10.3389/fcell.2021.627429

**Published:** 2021-02-09

**Authors:** Twan J. J. de Winter, Roeland Nusse

**Affiliations:** ^1^Faculty of Medicine, University Medical Centre Utrecht, Utrecht, Netherlands; ^2^Department of Developmental Biology, Howard Hughes Medical Institute, Stanford, CA, United States; ^3^School of Medicine, Institute for Stem Cell Biology and Regenerative Medicine, Stanford University, Stanford, CA, United States

**Keywords:** adipogenesis, Wnt signaling, mesenchymal stem cells, preadipocyte, osteogenesis, C/EBP, PPARγ

## Abstract

Mesenchymal stem cells (MSCs) give rise to adipocytes, osteocytes, and chondrocytes and reside in various tissues, including bone marrow and adipose tissue. The differentiation choices of MSCs are controlled by several signaling pathways, including the Wnt/β-catenin signaling. When MSCs undergo adipogenesis, they first differentiate into preadipocytes, a proliferative adipocyte precursor cell, after which they undergo terminal differentiation into mature adipocytes. These two steps are controlled by the Wnt/β-catenin pathway, in such a way that when signaling is abrogated, the next step in adipocyte differentiation can start. This sequence suggests that the main role of Wnt/β-catenin signaling is to suppress differentiation while increasing MSC and preadipocytes cell mass. During later steps of MSC differentiation, however, active Wnt signaling can promote osteogenesis instead of keeping the MSCs undifferentiated and proliferative. The exact mechanisms behind the various functions of Wnt signaling remain elusive, although recent research has revealed that during lineage commitment of MSCs into preadipocytes, Wnt signaling is inactivated by endogenous Wnt inhibitors. In part, this process is regulated by histone-modifying enzymes, which can lead to increased or decreased Wnt gene expression. The role of Wnt in adipogenesis, as well as in osteogenesis, has implications for metabolic diseases since Wnt signaling may serve as a therapeutic target.

## Introduction

Decades of research has established a main role of Wnt signaling in stem cell fate and control (Nusse, 2008; Van Camp et al., 2014). For example, Wnt/β-catenin signaling is among the main cell communication pathways in the intestinal stem cell niche in the crypts (Gehart and Clevers, 2019). Wnt signaling is also involved in differentiation and lineage fate decisions, as evinced in embryonic hematopoietic stem cell development (Richter et al., 2017). In mesenchymal stem cell (MSC) biology, activation of the β-catenin-dependent canonical Wnt pathway is essential to induce osteogenic differentiation (Kang et al., 2007). Over recent years, it has become clear that Wnt signaling also plays a major role in the process of adipogenesis, the differentiation of MSCs into mature fat cells, or adipocytes. Studies from Ross et al. and Bennet et al. demonstrated for the first time that autocrine Wnt expression suppresses terminal differentiation into mature adipocytes from the precursor preadipocytes (Ross et al., 2000; Bennett et al., 2002). Moreover, Wnt is also involved during the first stages of adipogenesis, when adipocyte commitment is at the expense of osteogenesis, the formation of bone cells (Han et al., 2019).

Adipose tissue is a potential source of easily accessible MSCs (Tsuji et al., 2014). Applications include the development of replacement therapies for bone, cartilage, and adipose tissues (Lazar et al., 2018). Likewise, MSCs are also used to treat other diseases unrelated to connective tissue dysfunction, due to their signaling and inflammatory mediating properties (Alfaro et al., 2011). Wnt effectors may be used as pharmaceutical targets for the treatment of Wnt-related metabolic diseases such as obesity, type 2 diabetes (T2D), and osteoporosis (Baron and Gori, 2018; Chen et al., 2018). A better understanding of the signaling routes during stem cell maintenance and differentiation is essential for utilization in tissue engineering and safe applications in patients. In this review, we aim at clarifying the role of Wnt signaling from MSCs until adipogenesis.

## Mesenchymal Stem Cells

MSCs are multipotent adult stem cells and are the progenitors of many connective tissue types, including bone, fat, cartilage, and muscle. Thus, MSCs have the ability to differentiate into adipocytes, osteocytes, chondrocytes, as well as myocytes and fibroblasts (Figure 1). The cells can be found in many adult tissues, including bone marrow (BM), and adipose tissue (Alfaro et al., 2011). MSCs cell populations are quite heterogeneous but they can be distinguished from each other by a set of positive and negative surface markers. The markers that multipotent MSCs typically express are CD13, CD29, CD44, CD63, CD73, CD90, and CD105 and they are negative for hematopoietic antigens CD14, CD31, and CD45 (Alfaro et al., 2011; Tsuji et al., 2014). MSCs are identified as having the ability to differentiate into bone, cartilage, and fat lineages both *in vitro* and *in vivo*. Primary MSCs can be isolated from tissues and can be cultured *in vitro*. Typically, the multipotency of primary isolated MSCs is tested by differentiation into the individual descendants, confirmed by Oil Red-O staining of neutral lipids for adipocytes, staining for mineralization for osteocytes, and staining for glycosaminoglycans for chondrocytes (Alfaro et al., 2011). After a number of passages cultured MSCs generally become senescent (Bork et al., 2010). Consequently, permanent MSC lines like the murine C3H10T1/2, are used experimentally (Tang et al., 2004). The heterogeneous nature of MSCs is also true for resident populations in tissues: while adipose-residing cells possess multi-lineage potential, they have greater adipogenic potential (Tsuji et al., 2014). Likewise, BM-MSCs are more biased to differentiate into an osteogenic lineage, in addition to forming BM-adipocytes (Tsuji et al., 2014; Bukowska et al., 2018).

**Figure 1:** Differentiation lineage potential of MSCs into bone (osteogenesis), adipose tissue (adipogenesis), cartilage (chondrogenesis), and muscle (myogenesis).

## Canonical and Non-Canonical WNT Signaling

The Wnt signaling pathways are a collective of signaling pathways activated by a family of Wnt proteins. The most commonly implicated Wnt pathway is through β-catenin, also termed the canonical Wnt pathway. Non-canonical systems include the planar cell polarity (PCP) and Wnt/Calcium pathways. Wnt signaling plays important roles during embryonic development as well as in adults (Nusse, 2008). When Wnt is not present, β-catenin, localized in the cytoplasm, is continuously degraded through the action of the “destruction complex.” This multiprotein complex consisting of scaffold protein axis inhibition protein (Axin), adenomatous polyposis coli (APC), casein kinase 1 (CK1), and glycogen synthase kinase 3 (GSK3), phosphorylates the N-terminus of β-catenin which is then recognized by β-Trcp, an E3 ubiquitin ligase subunit, followed by ubiquitination and subsequent proteasome degradation. Destruction of β-catenin prevents its nuclear localization. The signaling cascade of the Wnt pathway begins when one of the Wnt ligands binds to the receptor Frizzled (Fz) and its co-receptor low-density lipoprotein receptor-related protein 5 and 6 (LRP5/6). Once bound, this can recruit the scaffolding protein Disheveled (Dvl) to the receptor complex and after phosphorylation of LRP5/6, this recruits the destruction complex to the receptors, inhibiting the β-catenin phosphorylating activity. If β-catenin is active and stable, it translocates to the nucleus where it forms complexes with co-activators, such as transcription factor family DNA-bound T cell factor/lymphoid enhancer factor (TCF/LEF) (MacDonald et al., 2009). This transcription factor complex starts the expression of downstream targets genes, including Axin2, a Wnt signaling repressor (Leung et al., 2002). Several mechanisms are involved in endogenous inhibition of Wnt signaling.

Secreted Wnt inhibitors factors include Wnt inhibitor protein (WIF) and secreted Frizzled-related proteins (sFRPs). Dickkopf (DKK) is a secreted factor that binds and inhibits the LRP5/6 co-receptors (MacDonald et al., 2009). Other endogenous inhibitors, such as Axin2, act downstream of the Wnt signaling pathway (Leung et al., 2002).

## Adipogenesis and Preadipocytes

Adipose tissues fall into two distinct groups: the more common white adipose tissue (WAT; e.g., subcutaneous WAT and visceral WAT) and brown adipose tissue (BAT). These are both derived from adipose-residing MSCs and are generated in a stepwise differentiation program. MSCs first differentiate into an intermediate cell type called preadipocytes, during which the cells undergo growth arrest and mitotic clonal expansion (Lazar et al., 2018). Preadipocytes are proliferative, are presumably located near the vasculature in adipose tissues (Tsuji et al., 2014; Zhang et al., 2018) and have fibroblast-like morphology. Preadipocytes express the adipogenic transcription factors CCAAT-enhancer-binding protein β and δ (C/EBPβ/δ) and low but detectable levels of Peroxisome proliferator-activated receptor γ (PPARγ) (Park et al., 2004). In preadipocytes C/EBPβ is present in an inactive state and unable to start transcription of genes that initiate terminal differentiation (Park et al., 2004). PPARγ is an indispensable master regulator of the adipocyte transcriptional program. PPARγ expression is also required during the maintenance of mature adipocytes (Lee and Ge, 2014).

Terminal differentiation of preadipocytes into mature adipocytes can be triggered by pro-adipogenic signals (e.g., insulin; dexamethasone; 3-isobutyl-1-methylxanthine, IBMX; or bone morphogenetic proteins, BMPs), resulting in the upregulation of the adipogenic transcription factors PPARγ and C/EBPα (Tang et al., 2004; Wang et al., 2014). The differentiating cells morphologically change from a fibroblast-like morphology into a spherical shape with a single large lipid droplet (Lazar et al., 2018). Mature adipocytes are cells with metabolic and endocrine properties. These characteristics are initiated after activation of metabolic and adipogenic-specific genes, like fatty acid-binding protein 4 (FABP4), glucose transporter type 4 (GLUT4), leptin, and adiponectin. The differentiating cells assemble the machinery that mediates lipogenesis, the metabolic pathway that converts carbohydrates into triacylglycerols for storage. In addition, the cells become insulin sensitive, which is responsible for carbohydrate uptake (Cristancho and Lazar, 2011). Although the scope of this review is to discuss Wnt during adipogenesis, Wnt signaling also has notable roles in mature adipocytes, such as lipogenesis (Bagchi et al., 2020). A commonly used cell line for adipogenesis research is the mouse-derived permanent 3T3-L1 preadipocyte line. The cells can easily be grown *in vitro* and can be differentiated into a mature adipocyte phenotype (Bennett et al., 2002).

## Effects of WNT Function in Preadipocytes

In general, Wnt signaling is often associated with stem cell control and maintenance. Stem cells receive signaling cues from themselves or neighboring cells and can respond with the appropriate manner; self-renewal or differentiation (Nusse, 2008). Two decades ago Wnt10b was identified in preadipocytes as an important factor in cell maintenance and proliferation. Wnt10b is highly expressed in preadipocytes of both human and mouse origins (Ross et al., 2000; Bennett et al., 2002; Christodoulides et al., 2006). Later, Wnt10a and Wnt6 were also found to have similar control on stem cell maintenance (Cawthorn et al., 2012). *In vitro* studies have shown that blocking the Wnt pathway downstream of Wnt10b/10a/6 leads to spontaneous differentiation into mature adipocytes, and accordingly, overexpression of Wnt10b/10a/6 prevented adipogenesis (Ross et al., 2000; Bennett et al., 2002; Cawthorn et al., 2012). Genetically engineered mice that miss both alleles of *Wnt10b* have adipogenic as well as osteogenic abnormalities (Ross et al., 2000; Bennett et al., 2002; Stevens et al., 2010; Cawthorn et al., 2012). Perhaps the most compelling evidence that Wnt10b controls MSC and preadipocyte cell maintenance in mice is the progressive absence of adipogenic and osteogenic progenitors and premature adipogenesis/osteogenesis in Wnt10b-null mice (Stevens et al., 2010) Moreover, there is evidence that the expression of endogenous Wnt inhibitors (e.g., WT1 and sFRP1) in preadipocytes is significantly lower compared to mature adipocytes (Cho et al., 2019).

Wnt signaling impacts the expression of key transcription factors important in adipocyte differentiation, as has been shown by the MacDougald lab: active Wnt signaling in preadipocytes lowers RNA and protein levels of transcription factors C/EBPα and PPARγ, both needed for terminal differentiation. This suggests that Wnt signaling actively inhibits the expression of C/EBPα and PPARγ in preadipocytes (Ross et al., 2000; Bennett et al., 2002; Longo et al., 2004). The exact underlying mechanism of these effects was, until recently, poorly defined. However, a study by Xie et al. found that Wnt signaling through Axin2 directly inhibited the transcriptional activity of C/EBPβ (Figure 2) (Ross et al., 2000; Bennett et al., 2002; Longo et al., 2004; Xie et al., 2018). Active Wnt signaling in preadipocytes maintains the expression of Axin2. In the cytoplasm, Axin2 binds with the Wnt-related kinase GSK3β, which prevents GSK3β localization in the nucleus. GSK3β is mainly present in the cytoplasm, but can also be localized into the nucleus where it possesses kinase activity (Ross et al., 2000; Bennett et al., 2002; Longo et al., 2004; Shin et al., 2012; Xie et al., 2018). Given the fact that Axin1 and 2 are largely functional and structural similar (Chia and Costantini, 2005), it remains to be investigated why GSK3β is not retained in the cytoplasm by Axin1 during the Wnt off state. Without GSK3β in the nucleus C/EBPβ and Snail remain unphosphorylated, the absence of phosphorylation decreases the DNA binding activity of C/EBPβ and increases the stability of Snail (Park et al., 2004; Tang et al., 2005). Unphosphorylated C/EBPβ cannot start the expression of C/EBPα and PPARγ and stable Snail blocks PPARγ expression. Disruption of Wnt signaling leads to nuclear localization and phosphorylation activity of GSK3β, followed by the expression of C/EBPα and PPARγ mediated by active C/EBPβ (Xie et al., 2018). In turn, PPARγ binds to the Axin2 promoter and activates its transcription, leading to continuous canonical Wnt inhibition (Jho et al., 2002; Hu et al., 2015). Although Axin2 blocks PPARγ expression, PPARγ does not inhibit its own expression in a negative feedback loop. In 3T3-L1 cells, the expression of PPARγ peaks at day 6 of adipocyte differentiation and remains expressed even in mature adipocytes (Jitrapakdee et al., 2005). This could be explained by the fact that several transcription factors (e.g., C/EBPs, KLFs, etc.), induced at various time points of differentiation can directly activate gene expression of PPARγ and hereby maintaining its expression pattern (Jitrapakdee et al., 2005; Lee and Ge, 2014).

**Figure 2:** The mechanism of the inhibitory role of Wnt/β-catenin pathway in preadipocytes during adipogenesis. (Left) When in preadipocytes the canonical Wnt pathway is turned on by autocrine Wnt10b, this leads to nuclear localization of β-catenin in the nucleus, where it can bind with LEF/TCF. This transcription factor complex starts the expression of Axin2 and other genes related to stem cell maintenance and proliferation. Axin2 binds with GSK3β in the cytoplasm, thereby preventing migration into the nucleus. In this state, inactive C/EBPβ prevents the expression of transcription factors C/EBPα and PPARγ. Additionally, Snail inhibits the expression of C/EBPα. (Right) If the Wnt pathway is turned off this results in the start of terminal differentiation into mature adipocytes. Immediately preceding Wnt inactivation in preadipocytes, destruction of β-catenin in the cytoplasm by the destruction complex results in an absence of nuclear β-catenin. Without Axin2, GSK3β localizes into the nucleus where it phosphorylates Snail and C/EBPβ. Phosphorylation of Snail is accompanied by its degradation while phosphorylation of C/EBPβ renders its activation. These events start the expression of PPARγ C/EBPα, both crucial for initiating the final stage of adipogenesis. Changes in gene expression and epigenetic regulators prevent the production and secretion of endogenous Wnt ligands. Moreover, PPARγ starts the expression of Axin2, a Wnt signaling inhibiter.

## Epigenetic Regulation of WNT in Adipogenesis

Once Wnt signaling is inactivate in preadipocytes, the persistent Wnt expression has to be shut off. Recent research has shown that the control of enzymes involved in epigenetic regulation plays a role in this process. Histone acetyltransferases and histone methyltransferases are enzymes that modify lysine and arginine residues on histone proteins, by doing that they change the DNA accessibility, making genes more or less likely to be transcribed (Jing et al., 2018). Several studies suggest that this epigenetic regulation is involved in the way cells respond to Wnt signaling during adipogenesis. After activation of C/EBPβ during terminal differentiation, this transcription factor is able to start the transcription of lysine demethylase 5A (KDM5A), a transcriptional repressor. KDM5A knockdown by siRNAs resulted in the upregulation of anti-adipogenic Wnt6, so it is believed that the epigenetic changes caused by KDM5A after induction of adipogenesis inhibit the Wnt signaling pathway by preventing the expression of Wnt ligands (Guo et al., 2019).

Enhancer of zeste homolog 2 (EZH2) marks the promoters of *Wnt1/6/10a/10b* during adipocyte differentiation with the repressive epigenetic marker H3K27me3, thus reducing Wnt expression. EZH2 knockout blocks adipogenesis of brown preadipocytes, accompanied by significant upregulation of the Wnt genes. Moreover, these studies reported on a decrease of H3K27me3 on Wnt promoters and a global increase of the activating marker H3K27ac levels (Wang et al., 2010). Due to the changes of H3K27ac in EZH2 knockout cells, which can alter overall gene expression, the precise role of EZH2 remains unknown.

Additionally, the activity of epigenetic enzymes also affects how MSCs and preadipocytes respond to Wnt signaling. Histone Acetyltransferase GCN5 (GCN5), an enzyme that acetylates histone 3 on lysine 9 (H3K9ac), is known to prime the activation of Wnt genes, resulting in reduced adipogenesis (Jing et al., 2018). In BM-MSCs, GCN5 is able to prime transition of cells into an osteogenic lineage and to alter osteogenic activating signaling pathways (Zhang et al., 2016). A recent study by Sen et al. found that the histone methyltransferase activity of EZH2 activity could be responsible for keeping MSC in an undifferentiated state during Wnt signaling activation, since EZH2 knockdown in BM-MSCs resulted in osteogenesis (Sen et al., 2020). These findings emphasize that the epigenetic landscape of MSCs and preadipocytes has a regulatory role in the precise effect of Wnt signaling. The epigenetic enzymes change the likelihood of gene transcription, which is cell type-dependent. Therefore, in order to describe the role of Wnt signaling on heterogeneous cell populations such as MSCs and preadipocytes, it is required to have a better understanding of the underlying epigenetics.

## WNT Signaling During Adipogenesis

Since inhibition of the autocrine effect of Wnt10b leads to spontaneous adipocyte differentiation, it is widely believed that Wnt signaling inactivation is needed for differentiation (Figure 3). In fact, when 3T3-L1 cells are treated with the common terminal adipocyte differentiation protocol (methyl-isobutylxanthine, dexamethasone, and insulin) the cells have elevated levels of intracellular cAMP which leads to subsequent downregulation of Wnt10b expression (Bennett et al., 2002; Prestwich and MacDougald, 2007). Groucho family member transducin-like enhancer of split 3 (TLE3), a transcriptional coregulator, antagonizes TCF4 during terminal differentiation. This mechanism is speculated to prevent the expression of β-catenin-dependent Wnt target gene expression during differentiation (Villanueva et al., 2011). The antagonistic effect of pro-adipogenic factors on Wnt signaling is also seen in other signaling factors, including BMPs. These are members of the transforming growth factor β (TGF-β) signaling family and are essential molecules for triggering of differentiation of MSCs (Wang et al., 2014). BMP2 and BMP4 are known for their importance in the first step of adipogenesis. BMP2 mainly possesses pro-osteogenic properties but was also shown to be adipogenic. BMP4 is a known pro-adipogenic factor. BMP4 or 2 treatment in cultured murine C3H10T1/2 MSC cells differentiates these cells into a proliferating preadipocyte phenotype. Applying the terminal adipocyte differentiation protocol on BMP4-induced preadipocytes successfully generated mature adipocytes (Tang et al., 2004). Mechanistically BMPs act via SMAD1/5/8 proteins or an alternative pathway, via p38 mitogen-activated protein kinase (p38MAPK) (Wang et al., 2014). Lysyl oxidase (Lox) is a protein expressed downstream of p38MAPK and stimulates adipogenesis. Inhibition of Lox not only results in an absence of adipogenesis but also leads to an elevated activation of the Wnt signaling pathway and BMP4-induced osteogenesis (Jiang et al., 2018). These findings suggest that the on or off state of the canonical Wnt pathway determines the lineage potential during BMP-induced differentiation of MSCs. This is in line with the well-established required role of Wnt signaling activation during osteogenesis (Day et al., 2005; Hill et al., 2005).

**Figure 3:** The effect of canonical Wnt during the several stages of adipogenesis and early osteogenesis from MSCs.

Wnt5a and b, two Wnt proteins responsible for turning on non-canonical signaling have been described to have pro-adipogenic properties. Importantly, Wnt5a/b have a direct effect on the adipose transcription factors, since they are able to activate PPARγ (van Tienen et al., 2009). However, the effects of Wnt5a/b are not always consistent and unlike the canonical Wnt signaling pathway, the importance of non-canonical Wnts during adipogenesis *in vivo* is less established (Fuster et al., 2015). For instance, Wnt5a/b have a completely opposite effect in BM-MSCs compared to preadipocytes. In BM-MSCs they are anti-adipogenic and have the potential to induce osteogenesis by upregulation of osteogenic master regulator Runt-related transcription factor 2 (Runx2) (Kitagawa et al., 2007). In addition, the role of Wnt5a is dose-dependent in rat MSCs and preadipocytes, lower concentrations have been shown to prevent adipogenesis and higher concentrations are pro-adipogenic, via an anti-β-catenin and Wnt/PCP-independent manner (Tang et al., 2004; Kitagawa et al., 2007). The multifactorial role is related to which type of signaling pathways are activated by Wnt5a/b proteins. For instance, Park and colleagues found an alternative Wnt signaling mechanism independent of the canonical Wnt pathway. This signaling pathway, named Wnt-YAP/TAZ, interacts with the non-canonical PCP/Wnt pathway and have Yes-associated proteins (YAP) and transcriptional coactivator with PDZ-binding motif (TAZ) as downstream effectors (Park et al., 2015). Wnt5a/b are agonists of Wnt-YAP/TAZ signaling and there is evidence that it can initiate terminal adipocyte differentiation (Park et al., 2015). To activate this pathway, Wnt5a/b bind to the Fz receptor, and the tyrosine kinase-like orphan receptor 1 and 2 (ROR1/2) have to act as co-receptors (Ackers and Malgor, 2018). MSCs from adipose tissue have been shown to contain a significantly higher population of ROR2 positive cells compared to BM-MSCs (Dickinson et al., 2017). Consequently, this could point out that the effect of non-canonical Wnt is cell type-dependent.

## WNT/β-Catenin in Early Osteogenesis

The formation of bone cells (or osteogenesis), happens at the expense of adipocyte differentiation, and this bifurcation is regulated by Wnt signaling. Two distinct mechanisms are involved in skeletal bone development, intramembranous and endochondral ossification. The first is characterized by direct formation of osteoblasts while the latter proceeds through an intermediate step of chondrocytes (Day et al., 2005). During the formation of intramembranous bone, MSCs directly differentiate into heterogenous osteoblast precursors which can later develop into osteocytes (Franz-Odendaal et al., 2006). The differentiation program is launched when the cells start expressing the osteogenic transcription factors Runx2 and SP7/Osterix (Komori, 2011). Runx2 is for example responsible for the expression of bone matrix proteins and Osterix for the upregulation of proteins initiating mineralization (Renn and Winkler, 2009; Komori, 2010). It is well-established that Wnt signaling can directly promote this differentiation process. Activated β-catenin starts the expression and activation of Runx2 which then results in the expression of transcription factors Osterix and TCF7. Noteworthy, Runx2 expression can also be induced by other signals such as fibroblast growth factor or Hedgehog (Komori, 2011). Mice with a conditional deletion of β-catenin in preosteoblasts exhibit a complete block of osteoblast differentiation, but these cells still expressed Runx2 (Day et al., 2005; Hill et al., 2005). This means that the induction of Runx2 expression does not depend on Wnt signaling, but that the signaling cascade is vital to proceed osteogenesis. A recent study found that a novel regulator of the Wnt pathway, Z-DNA-binding protein 1 (ZBP1), formed a positive feedback loop with the Wnt signaling pathway that could inhibit adipogenesis and promote osteogenesis. Moreover, ZBP1 was required for Wnt signaling in MSCs, indicating that ZBP1 could play a role in lineage specification of MSCs (Zhao et al., 2020).

## The Role of WNT During *in vitro* MSC Expansion and Regenerative Medicine (RM)

MSCs can truly be beneficial for use in RM since there are many clinical applications for the cells, including bone, fat, and cartilage graft development for (auto)transplantation. Although isolated human MSCs are self-renewing stem cells, they have limited doubling potential when cultured *in vitro*. Long term culture of MSCs renders the cells senescent, and the cells stop proliferating (Liu et al., 2020). This is a major hurdle, since expansion might be needed to collect enough cells to create an MSC-derived graft (Liu et al., 2020). Signaling factors such as FGF, have the potential to stimulate MSC expansion and prevent them from becoming senescent (Tsutsumi et al., 2001; Bork et al., 2010). Likewise, active β-catenin in MSCs has been associated with increased proliferation without altering its potential to differentiate into adipocytes, osteocytes, or chondrocytes. Treatment of murine C3H10T1/2 cells with β-catenin agonist, 6-bromoindirubin-3′-oxime (BIO), showed that besides significant increase of proliferation, the cells exhibited higher levels of expression of pluripotency genes SRY-box 2 (Sox2), Nanog, octamer-binding transcription factor 4 (Oct4), and Cyclin D1 (Hoffman and Benoit, 2015). In MSCs, these markers have been demonstrated to have a direct effect on maintaining the undifferentiated state as well as promoting proliferation (Tsai and Hung, 2012). MSCs extracted from different locations express several Wnt ligands, and endogenous Wnt signaling is required for stem cell maintenance (Etheridge et al., 2004; Tantrawatpan et al., 2013; Jothimani et al., 2020). Thus, this suggests that the canonical Wnt pathway mediates the stemness as well as osteogenesis in an intricate balance. However, more research has to be carried out to establish this underlying mechanism and how to apply this *in vitro*.

## Impaired WNT Signaling in MSCs

Impaired Wnt signaling can lead to disease, and this is also true for mesenchymal tissues. Since mesenchymal tissue types are constantly renewed (Alfaro et al., 2011), impaired signaling can have significant effects on metabolism, as seen in osteoporosis, T2D, and obesity (Baron and Kneissel, 2013; Chen et al., 2018). One example of overly active Wnt signaling in adipose tissue is seen in T2D patients with a mutation in the transcription factor 7-like 2 gene (*TCF7L2*) (Chen et al., 2018), a transcriptional repressor of the Wnt signaling pathway (Mandal et al., 2017). *In vivo* experiments with inactive mutations of TCF7L2 results in impaired adipogenesis characterized by increased subcutaneous adipose tissue mass, adipocyte hypertrophy, and inflammation. All mechanisms that are manifested when there is an excess of lipids. Moreover, this was accompanied by whole-body glucose intolerance and hepatic insulin resistance, a T2D hallmark (Kahn et al., 2006; Jo et al., 2009; Chen et al., 2018). On the other hand, a decrease in Wnt activity can also be detrimental, as seen in osteoporosis. Osteoporosis is a bone disease characterized by lowered bone density and increased bone fragility. Patients suffering from this disease have diminished osteogenesis and the Wnt signaling pathways are shown to be responsible. More specifically, loss-of-function mutations of the co-receptors LRP5/6 were identified as the cause (Baron and Kneissel, 2013). Increased BM adipose tissue (BMAT), a special type of adipose tissue distinct from WAT or BAT naturally residing in BM (Bukowska et al., 2018), is also related to osteoporosis. The lineage potential of MSCs from patients with osteoporosis was more biased toward differentiation into adipocytes and signaling from BMAT was shown to promote adipogenesis of BM-MSCs (Astudillo et al., 2008). Wnt and its downstream effectors could serve as potential therapeutic targets (Hoeppner et al., 2009).

## Concluding Remarks

Adipogenesis, the process of the formation of adipocytes from MSCs, is tightly regulated by signaling pathways. The Wnt signaling pathways are among these and have been proven to be crucial for MSC lineage specification. It is widely documented that canonical Wnt signaling regulates several steps in this differentiation process, but the precise underlying mechanisms remain poorly understood. In recent years, MSCs have been shown to be promising for use in regenerative medicine (Hoeppner et al., 2009; Alfaro et al., 2011).

In adipose tissue, Wnt signaling promotes stem cell maintenance of preadipocytes. The stem cell niche of preadipocytes, however, does not solely consist of preadipocytes and adipocytes. Other cell types that reside in the cell type niche are fibroblasts, immune cells, endothelial cells, and a small fraction of MSCs. Preadipocytes can be found in the stromal vascular fraction of adipose tissue and this is believed to be in close proximity of the blood vessels (Tsuji et al., 2014; Zhang et al., 2018). Secretion of signaling factors by some of these neighboring cells was shown to be essential in the mediation of adipogenesis (Zhang et al., 2018; Sebo and Rodeheffer, 2019). It remains unclear if these other cell types also express Wnt ligands, but autocrine action of Wnt10b/10a/6 by preadipocytes is believed to be the main source (Ross et al., 2000; Bennett et al., 2002; Cawthorn et al., 2012).

A limitation of many studies related to adipogenesis and MSCs biology is the use of non-human permanent cell lines 3T3-L1 and C3H10T1/2 (Ross et al., 2000; Longo et al., 2004; Tang et al., 2004), although they provide consistency across experiments, which would be difficult with isolated human MSCs and preadipocytes. These permanent cell line do not faithfully represent the highly heterogeneous nature of MSCs, however. Primary cultures of MSCs should be included as well, but culturing these cells has been proven difficult (Bork et al., 2010).

In conclusion, Wnt signaling mainly plays a role in suppressing adipogenesis during several stages of differentiation. It seems that the main role of suppression is to increase the MSC and preadipocytes cell mass. Epigenetic and transcriptional regulators have a significant impact on this process, but it is still poorly understood how transcriptional regulation and Wnt signaling interact during adipogenesis.

## Author Contributions

TW performed the literature review, analyzed and interpreted the findings, and wrote the manuscript. RN supervised the writing process and edited the manuscript. All authors contributed to the article and approved the submitted version.

## Conflict of Interest

The authors declare that the research was conducted in the absence of any commercial or financial relationships that could be construed as a potential conflict of interest.
